# The Anticancer Potential of Chlorine Dioxide in Small-Cell Lung Cancer Cells

**DOI:** 10.7759/cureus.29989

**Published:** 2022-10-06

**Authors:** Salih Zeki Yıldız, Cemil Bilir, Gamze Guney Eskiler, Filiz Bilir

**Affiliations:** 1 Department of Chemistry, Faculty of Arts and Sciences, Sakarya University, Sakarya, TUR; 2 Medical Oncology, Istinye University, VM Medical Park Pendik Hospital, Istanbul, TUR; 3 Department of Medical Biology, Faculty of Medicine, Sakarya University, Sakarya, TUR; 4 Department of Gynecologic Oncology, Faculty of Medicine, Kocaeli University, Kocaeli, TUR

**Keywords:** small-cell lung cancer, anticancer, dms114 cell line, apoptosis, chlorine dioxide

## Abstract

Background

Chlorine dioxide (ClO_2_) is an effective disinfectant consisting of oxygen, chloride, and potassium. Because of its high oxidative capacity, ClO_2_ exerts antimicrobial, antiviral, and antifungal effects. However, its anticancer effects remain to be elucidated.

Methodology

The anticancer activity of CIO_2_ was assessed on DMS114 small-cell lung cancer (SCLC) cells and human umbilical vein endothelial cells (HUVEC) as control by WST-1, Annexin V, cell cycle analysis, and acridine orange staining. We for the first time investigated the possible therapeutic effects of long-term stabilized ClO_2_ solution (LTSCD).

Results

Our preliminary findings showed that LTSCD significantly inhibited the proliferation of SCLC cells (p < 0.01) with less toxicity in HUVEC cells. Additionally, LTSCD induced apoptotic cell death in SCLC cells through nuclear blebbing and vacuolar formation. However, LTSCD treatment did not induce cell cycle arrest in both cell lines.

Conclusions

LTSCD can be a therapeutic potential for the treatment of SCLC. However, further investigations are required to assess the LTSCD-induced cell death in SCLC both in vitro and in vivo.

## Introduction

Small-cell lung cancer (SCLC) comprises nearly 15% of all lung cancer cases globally, with 2.21 million individuals diagnosed with lung cancer in 2020. Patients with SCLC show poor prognosis with a median overall survival (OS) of approximately 12-20 months due to late detection and rapid tumor growth. In the treatment of SCLC, surgery, first-line standard chemotherapy (etoposide or irinotecan with platinum combination), and prophylactic cerebral irradiation are used. Additionally, some drugs are used for second-line treatment of SCLC. However, the majority of patients develop resistance to current treatment options and metastases in additional sites [1-4]. Therefore, alternative treatment strategies are urgently needed to obtain better treatment responses and improve the survival and outcomes of patients with SCLC.

Aqueous chlorine dioxide (ClO_2_) is an effective disinfectant and a water purifier and is used in mouth rinses and surface disinfectants. ClO_2_ consists of oxygen, chloride, and potassium, and its action depends on the release of nascent oxygen during the action. Therefore, ClO_2_ exerts high oxidative capacity and biocidal activity, making it a non-toxic, antimicrobial, antiviral, and antifungal agent. ClO_2_ accelerates wound healing, especially burns, by inducing cyclic GMP production through the induction of the guanylate cyclase enzyme [5-7]. However, few studies have investigated the anticancer activity of ClO_2_ in cancer treatment [8,9]. Indeed, ClO_2_ potentially inhibits the proliferation of cancer cells by inducing reactive oxygen species (ROS) production. In the study by Schwartz (2017), ClO_2_ treatment reduced the intracellular pH of cancer cells and improved two patient (pancreas and prostate cancer) outcomes [8]. Additionally, Kim et al. (2016) reported that ClO_2_ inhibits the proliferation of MCF-7 and MDA-MB-231 breast cancer cells as well as LoVo, HCT-116, and SW-480 colon cancer cells via the production of ROS [9]. Therefore, further investigations are required to evaluate the underlying molecular mechanism of ClO_2_-mediated anticancer effects on different types of cancer. In this context, this study aimed to investigate the cytotoxic and apoptotic effects of long-term stabilized ClO_2_ solution (LTSCD) on SCLC cancer cells in vitro.

## Materials and methods

The preparation of LTSCD

All reagents were purchased from Merck and Sigma-Aldrich. Analytical reagent-grade chemicals and distilled-deionized water were used throughout the study. The sodium chlorite was supplied as food grade 32% solution by Turoski Kimyevi Maddeler, Kocaeli, Turkey. Rhodamine B (RhB) was used as a fluorescent dye to determine the ClO_2 _concentration in the prepared solutions by a cross-checking approach using a fluorimeter and ultraviolet-visible (UV-Vis) spectrometer. Electronic spectra were recorded on a Shimadzu UV-2600 Pc-spectrophotometer with a quartz cell of 1 cm. Fluorescence excitation and emission spectra were recorded on a Varian Eclipse spectrofluorometer using 1 cm pathlength cuvettes at room temperature.

To prolong the shelf life, LTSCD was configured as a two-component product consisting of B for the base component and A for the activator. The ingredients of the components are listed in Table 1. The activated LTSCD could be prepared from the components as given in the following and used for a while.

**Table 1:** Ingredients of A and B used for the preparation of LTSCD. LTSCD: long-term stabilized ClO_2_ solution

B	A
16.5 g sodium chlorite (32% solution)	6.2 g sodium bisulphate
1.6 g sodium carbonate	19.4 g Sodium persulfate
481.9 g DI water	6.74 g citric acid
Total amount 500 g	677.5 g DI water
	Total amount 100 g

Component B was added to an amber-colored 750 mL polytetrafluoroethylene (PET) bottle, which was inert enough for the intended chemical and safer for the accident. Concentrated sulfuric acid (conc. H_2_SO_4_) (1.5 mL) was added to the bottle and the mouth was capped. The slightly acidified B mixture was allowed to stand for five minutes for activation. Subsequently, component A was added to the prepared mixture in a fume hood. The final mixture was allowed to stand for 24 hours and slightly covered for the removal of the generated gases and sufficient stabilization. The prepared LTSCD was stable for five months and could be used for three months in such studies safely. The concentration of the prepared LTSCD was 3000 ppm. However, it was diluted to 500 ppm and used as a stock solution to prolong the stability period. The stock solution was stored in cool (4°C) and dark conditions and used to prepare a diluted application solution (containing 50 mg/L ClO_2_). For the freshly prepared or longer-stayed LTSCD solutions, it was recommended to control the concentrations by cross-checking using a UV-Vis spectrometer and fluorimeter, respectively.

Cell culture and cytotoxicity analysis

DMS114 cells and human umbilical vein endothelial cells (HUVEC) were obtained from ATCC and cultured in Dulbecco’s modified eagle medium (DMEM) medium supplemented with 10% fetal bovine serum (FBS) and 1% penicillin-streptomycin in a humidified incubator at 37°C. To determine the cytotoxicity of LTSCD in the cells, we conducted WST-1 analysis. The cells were exposed to different concentrations (0.1-10 mg/L) of LTSCD for 24 and 48 hours. Following incubation, the viability of the cells was measured using WST-1 dye by a multi-plate reader at 450 nm.

Annexin V and cell cycle analysis

ClO_2_-mediated apoptotic effects were analyzed by Annexin V and cell cycle analysis. The cells were treated with the most effective concentration of LTSCD for 48 hours. Following treatment, the cells were re-suspended and washed with phosphate-buffered saline (PBS). Afterward, the cells were stained with Annexin V and 7-AAD dye for Annexin V analysis. For cell cycle analysis, the cells were fixed with 70% cold ethanol for two to three hours and stained with cell cycle dye. After staining, the cells were analyzed by a Muse Cell Analyzer.

Acridine orange (AO) staining

To observe ClO_2_-induced apoptotic death, the cells were stained with AO. Following treatment with 1 and 5 mg/L LTSCD for 48 hours, the cells were fixed with 4% paraformaldehyde and stained with 1 mg AO dye. Following incubation for 30 minutes, the cells were washed with PBS and visualized through an EVOS Cell Imaging Station.

Statistical analysis

SPSS version 22 (IBM Corp., Armonk, NY, USA) was used for statistical comparison. To compare groups, a one-way analysis of variance post-Tukey analysis was used. P-values of <0.05 were considered significant.

## Results

Evaluation of LTSCD anticancer potential in DMS114 cells

To assess ClO_2_-mediated anticancer activity, we performed WST-1 analysis. As shown in Figure 1, the viability of DMS114 cells was significantly reduced in a dose-dependent manner (p < 0.01). The percentage of DMS114 cells was 96.3 ± 0.6%, 97.7 ± 0.7%, 88.7 ± 1.7%, 49.3 ± 2.5%, and 44.7 ± 0.4% at 0.1, 0.5, 1, 5, and 10 mg/L, respectively, for 24 hours. Furthermore, the viability of DMS114 considerably reduced to 66.0 ± 3.1%, 43.2 ± 1.5%, and 46.4 ± 1.6% after treatment with 1, 5, and 10 mg/L ClO_2_, respectively, for 48 hours. In HUVEC control cells, a 19.7 ± 2.2% and 25.5 ± 1.0% decrease was observed at 1 and 5 mg/L, respectively, for 48 hours. Therefore, LTSCD treatment did not result in a significant toxic effect on HUVEC cells and inhibited SCLC cell proliferation.

**Figure 1:** The viability of DMS114 and HUVEC cells after treatment with different concentrations of LTSCD for 24 and 48 hours by WST-1 analysis (p < 0.05*, p < 0.01**). HUVEC: human umbilical vein endothelial cells; LTSCD: long-term stabilized ClO_2_ solution

Evaluation of the apoptotic effects of LTSCD on DMS114 cells

We selected the most effective concentration (1 and 5 mg/L for 48 hours) of LTSCD according to WST-1 analysis. LTSCD treatment induced early apoptotic cell death, particularly in DMS114 cells, as shown in Figure 2. Following incubation with 1 and 5 mg/L LTSCD, total apoptotic death rate significantly increased to 37.2 ± 1.2% and 49.6 ± 0.8%, respectively, in DMS114 cells (p < 0.01), whereas 18.8 ± 0.5% and 27.6 ± 0.6% apoptotic deaths were detected in HUVEC cells, respectively, for 48 hours. Furthermore, ClO_2_-mediated apoptotic effects were also verified by AO staining (Figure 2B). Particularly, nuclear blebbing and vacuolar formation were observed in DMS114 cells at 5 mg/L for 48 hours. On the other hand, the morphology of HUVEC cells treated with LTSCD was similar to the control group. Additionally, LTSCD treatment induced the G2/M phase in DMS114 cells at 1 mg/L. However, LTSCD treatment did not induce cell cycle arrest in HUVEC cells due to less toxicity (Figure 3).

**Figure 2:** LTSCD-induced apoptotic effects evaluated by Annexin V analysis and AO staining. (A) The histograms of Annexin V analysis in (a) DMS114 and (b) HUVEC cells. (B) Statistical comparison of ClO_2_-induced early and late apoptotic death in the cells. (C) The images of (a) DMS114 and (b) HUVEC cells following treatment with 1 and 5 mg/L LTSCD for 48 hours (p < 0.05*, p < 0.01**). HUVEC: human umbilical vein endothelial cells; LTSCD: long-term stabilized ClO_2_ solution; AO: acridine orange

**Figure 3:** The cell cycle effects of LTSCD on (a) DMS114 and (b) HUVEC cells. (A) Histograms of cell cycle results. (B) Statistical comparison of the percentage of cells in G0/G1, S, and G2/M arrest following incubation with 1 and 5 mg/L of LTSCD (p < 0.05*, p < 0.01**). HUVEC: human umbilical vein endothelial cells; LTSCD: long-term stabilized ClO_2_ solution

## Discussion

This study showed that LTSCD exerted anticancer activity in SCLC cells through apoptotic cell death and G2/M arrest with less toxicity in HUVEC control cells. In the literature, the antibacterial, antiviral, and antifungal properties of ClO_2_ have been investigated due to its higher water solubility [10,11]. Recent studies have shown that ClO_2_ prevents the recombinant spike protein of severe acute respiratory syndrome coronavirus 2 by attaching to its receptor, angiotensin-converting enzyme 2 [12,13]. Additionally, ClO_2_ interacts with one or more cysteine, tyrosine, or tryptophan amino acid residues of the spike proteins in enveloped viruses and also attaches to the viral DNA of non-enveloped viruses [14,15]. However, the concentration, exposure time, pH, and temperature affect the antiviral and antimicrobial effects of ClO_2_ [16-18].

Furthermore, CIO_2_ interacts with aromatic amino acids and leads to the oxidization of the proteins, and binds to DNA or RNA [19,20]. In this context, Kim et al. (2016) evaluated the antiviral and anticancer effects of CIO_2_ and reported that CIO_2_ significantly inhibits breast and colon cancer cell proliferation due to possibly inducing ROS [9]. Another possible mechanism of CIO_2_-induced cytotoxicity is that CIO_2_ can oxidize polyamines, and these oxidative molecules, hydrogen peroxide and aldehydes, are extremely toxic to cancer cells. Furthermore, the increased hydrogen peroxide generated by oxidation can induce apoptosis, pyknosis, and necrosis. Therefore, CIO_2_-mediated oxidation causes cell death of cancer cells by endogenous hydrogen peroxide [21,22]. In our study, we showed that LTSCD considerably inhibited the proliferation of DMS114 cells with less toxicity in HUVEC cells. Additionally, LTSCD induced apoptosis with nuclear blebbing and G2/M arrest in DMS114 cells. However, dose-dependent G2/M arrest slightly increased in DMS114 cells. The oxidative stress and elevated ROS level induce the DNA damage response, leading to cell cycle arrest and causing apoptotic cell death [23]. However, imbalanced ROS levels and DNA damage overwhelm the DNA damage repair mechanism and cause exit from the cell cycle. Therefore, excessive damage leads to the exit cell cycle without triggering the cell cycle checkpoints and develops resistance despite apoptosis [23,24]. Therefore, further investigations should be conducted to elucidate the underlying mechanism of LTSCD-induced apoptosis and its association with the cell cycle.

This study has some limitations. This is the first study evaluating CIO_2_ efficacy in SCLC cells. Therefore, we did not compare its effect with any other chemotherapeutic drug. Second, we did not evaluate the underlying molecular mechanisms of LTSCD-induced apoptosis in vitro and in vivo. Therefore, we designed this study as preliminary research, and further investigations are needed to assess the anticancer activity of LTSCD in different types of cancer in line with these novel findings.

## Conclusions

LTSCD has anticancer effects on SCLC cells with less toxicity in HUVEC cells. Further research should be designed to assess the extensive mechanisms of LTSCD-induced cell death for the treatment of SCLC.
